The article "Ephedra alata subsp. alenda (Ephedraceae) leaf extracts: phytochemical screening, anti-diabetic, anti-obesity and anti-toxic activities on diabetic-induced liver-kidney-testes toxicities and inhibition of α-amylase and lipase enzymes" was retracted in 2024. Reasons: concerns about the data; concerns about a third party's involvement.

# *Ephedra alata* subsp. alenda (Ephedraceae) leaf extracts: phytochemical screening, anti-diabetic, anti-obesity and anti-toxic activities on diabetic-induced liver-kidney-testes toxicities and inhibition of α-amylase and lipase enzymes

**DOI:** 10.1016/j.heliyon.2022.e11954

**Published:** 2022-11-29

**Authors:** Saber Abdelkader Saidi, Turki M. Al-Shaikh, Othman A. Alghamdi, Khaled Hamden

**Affiliations:** a Department of Biology, College of Sciences and Arts-Khulis, University of Jeddah, Jeddah, Saudi Arabia; b Department of Biological Sciences, College of Science, University of Jeddah, Jeddah, Saudi Arabia; c Laboratory of Bioresources: Integrative Biology and Exploiting, Higher Institute of Biotechnology of Monastir, University of Monastir, Tunisia

**Keywords:** *Ephedra alata*, Obesity, Type 2 diabetes, Liver, Kidney, Testes

## Abstract

The study evaluated the phytochemical composition of *Ephedra alata* and its effects on α-amylase and lipase enzymes and diabetic-induced liver-kidney-testes toxicities to determine the anti-diabetic, anti-obesity, and anti-toxic potentials of the plant. Obesity was induced by a high-fat and fructose diet (HFFD). Various compounds were identified and quantified: cafeic acid, apigenin 7-O-glucoside, apigenin, rutin, luteolin 7-O-glucoside, p-Coumaric acid and others in EA aqueous extract (EAWE). *In vitro*, this study showed that EAWE strongly inhibited lipase activity as compared to EA methanol (EAME) and ethyl acetate EA extracts (EAEE). In obese rats, the supplementation of EAWE inhibited significantly (P < 0.01) intestinal and pancreatic lipase activity by 35 and 36% respectively. This decrease in lipid digestive enzyme activity caused a significant (P < 0.05) reduce in the weight gain by 12.7% and significant (P < 0.05) decrease in the serum lipid rate as total cholesterol (TC), low-density lipoprotein cholesterol (LDL-C) and high-density lipoprotein cholesterol (HDL-C). Moreover, the supplementation of EAWE to obese rats reduced the activity of α-amylase in the small intestine and pancreas by 26 and 31% respectively (P < 0.01) and consequently decreases in serum glucose level by 20.8% (P < 0.05). In addition, administration of EAWE in type 2 diabetes protected from obesity induced liver, kidney and testes alterations. The potent protective effect EAWE may be influenced by the diversity of phenolic compounds. therefore, this study showed in the first time that EAWE are efficient for the prevention and the amelioration of obesity, hyperglycemia, and various organs toxicities.

## 1 Introduction

Obesity is a metabolic disease characterized by increased blood glucose and sugars, lipids, and proteins metabolisms disorders. This disease contributes to various perturbations and diseases, such as type 2 diabetes, hypertension, heart diseases, cancers and various others diseases [1,2]. Statistical studies by the WHO have showing in 2016, around 2 billion adults were overweight, and more than more than half a billion, were obese worldwide [3]. In addition, type 2 diabetes causes various diseases and perturbations as hypertension, arteriosclerosis and cardiovascular diseases. One therapeutic approach for the prevention of obesity and type2 diabetes is to retard the absorption of glucose and fatty acid by the inhibition of α-amylase and lipase in the intestine [[4], [5], [6], [7], [8], [9], [10]]. Synthetic drugs as orlistat and acarbose are an intestinal α-amylase and lipase inhibitors, but caused various adverse effects such as gastrointestinal symptoms, abdominal discomfort and flatulence [11].

The article "Ephedra alata subsp. alenda (Ephedraceae) leaf extracts: phytochemical screening, anti-diabetic, anti-obesity and anti-toxic activities on diabetic-induced liver-kidney-testes toxicities and inhibition of α-amylase and lipase enzymes" was retracted in 2024. Reasons: concerns about the data; concerns about a third party's involvement.

Medicinal plants have always been important in many fields worldwide and contain certain contain various types of bioactive compounds with multiple therapeutics effects. In fact, plant phenolics drugs have been used for the treatment and prevention of multiple human diseases including diabetes, cancer, hypertension, and others [[12], [13], [14], [15], [16], [17], [18]]. *Ephedra alata* was an important source of various bio-actives drugs such glycosides, flavonoids, phenolic compounds, and alkaloids. Previous studies reported have reported that this plant exert identical biological activities as antibacterial, liver function protection, prevention of cardiovascular diseases, and prevention and amelioration of cancer [[17], [18], [19], [20], [21], [22], [23], [24], [25]]. A number of natural products possess the ability to prevent obesity by digestive enzymes as lipase and α-amylase [6,[26], [27], [28]]. In fact, the inhibition of lipase and α-amylase by natural products aids gastric emptying, which are useful in the treatment of obesity, diabetes and hyperglycaemia induced various organs toxicities without adverse effects [5,10,29,30]. No study has, however, been provided on the phytochemical composition of *Ephedra alata* (EA) water, methanol and ethyl acetate extracts and their effect on lipase and α-amylase activities in HFFD-induced obesity and insulin resistance. Accordingly, this study evaluated the action of the administration of EA aqueous extract (EAWE) to obese rats by gastric gavage route on the lipase and α-amylase activities, insulin resistance and glycogen level, and type 2 diabetes induced various organs toxicities.

## 2 Materials and methods

### 2.1 Plant materials

#### 2.1.1 *Ephedra alata* collection, preparation, and extraction

Fresh harvested plant material (*Ephedra alata* subsp. Alenda) was collected from Gafsa (Tunisia) in April 2020 (http://maps.google. 4.67919441906935,10.723443478345871), and identified as *Ephedra alata* subsp. Alenda (Ephedraceae) by a botanist at Sfax University, Faculty of Sciences of Sfax. A voucher specimen (NO.Ea 20–23) has been deposited in our laboratory. The leaves were dried at room temperature using a convection oven at 35 °C for three days. EA leaves were grinded into fine powder using an electric blender (moulinex, France). Each powdered leaves (100 g) were extracted with methanol or ethyl-acetate with soxhlet technique for 9h. The EAME and EAEA extracts were dried at 45 °C by rotavap. The EAWE was obtained by boiling 100g of EA powdered leaves in 500 ml distilled water during 20 min. The extract was filtered and lyophilized (−85 °C, 72 h). EAWE, EAME and EAEA were kept at -80 °C until phytochemical and biologicals evaluations [31].

The article "Ephedra alata subsp. alenda (Ephedraceae) leaf extracts: phytochemical screening, anti-diabetic, anti-obesity and anti-toxic activities on diabetic-induced liver-kidney-testes toxicities and inhibition of α-amylase and lipase enzymes" was retracted in 2024. Reasons: concerns about the data; concerns about a third party's involvement.

#### 2.1.2 High-performance liquid chromatography with diode array detection (HPLC- DAD) analysis

The detection and the quantification of EA extracts phenolic compounds was determined using HPLC- DAD system (Agilent, USA) by a diode array detector (DAD). The EA phenolic compounds separation was realized by C18 column at 40 °C. The mobile phase is formed of 0.1% formic acid in water (A) versus 0.1% formic acid in acetonitrile (B) during running time of 60 min. The injection volume was 10 μL; and the EA extracts phenolic compounds will detect by comparing the relative elution order and UV spectra [25]. The identification of each peak was established by LC–MS, performed on an Agilent 1100 LC system.

### 2.2 In vitro experiments

#### 2.2.1 α-amylase activity inhibition in vitro

α-amylase inhibition activity was determined according of the method described previously [26]. 0.5 mg of α-amylase from porcine pancreas (Sigma, ref A4268) has been dissolved in 1 ml phosphate buffer (20-mM, pH, 6.9). The mixture composed of 1 ml of EAWE, EAME or EAEA and 1 ml of α-amylase mixture (12 U/ml). The reaction medium incubated at 37 °C during 15 min and then 1 ml of starch (0.5%) was added to the mixture and reserved at 37 °C for 15 min. The reaction arrested by addition 2 ml dinitrosalicylic acid (DNS) was supplemented. Then cooled and measured absorbance at 565 nm. All the measurements including control and background samples were conducted in triplicate.

#### 2.2.2 Lipase activity determination in vitro

The lipase activity was measured by the mixture of 1 ml of extract and 1 ml of lipase from porcine pancreas (Sigma, ref L3126) at concentration 0.1 mg/ml mixed in a potassium phosphate buffer (0.1mM, pH 6.0). The reaction mixture was re-incubated for 10 min at 37 °C. After adding 0.1ml p-NPP substrate, the mixture incubated at 37 °C during 15 min, and the optical density was noted at 410 nm [26]. The inhibition activity was determined by formula: % activity = (A_C_-A_S_/A_C_) x100.

The article "Ephedra alata subsp. alenda (Ephedraceae) leaf extracts: phytochemical screening, anti-diabetic, anti-obesity and anti-toxic activities on diabetic-induced liver-kidney-testes toxicities and inhibition of α-amylase and lipase enzymes" was retracted in 2024. Reasons: concerns about the data; concerns about a third party's involvement.

Ac and As: optical density of control and sample at 410 nm respectively. Each experiment was performed in triplets**.**

### 2.3 In vivo experiments

#### 2.3.1 Animals

26 Male *Wistar* rats weighing (176g ± 17) and aged 12 weeks were used for this study. The animal study protocol was also approved by the Ethics Committee of Monastir University and was conducted following international guidelines for animal experimentation (Approval No. MU-86/609/EEC). The rats were preserved in separate stainless-steel wire mesh cages. Food and drinking water were available ad libitum with environmental conditions: humidity of 55 ± 5%, room laboratory (25–30 °C), and under 12-hour dark and 12-hour light.

#### 2.3.2 Induction of obesity

The study was conducted according of previous study [26]. The HFF-diet was constituted of 60% of standard diet, 11,69% sheep fats, 10% fructose and 0.5% cholic acid as described by previous study [26]. Rats were fed ad libitum either a standard chow. A weekly control of solid and liquid intake was performed. The induction of obesity and type 2 diabetes were achieved by a important increase in body weight and blood glucose level as compared to normal rats.

#### 2.3.3 Experimental design and procedure

32 rats were randomly allocated to 8 experimental groups as follow: Group 1, control rats fed on a normal diet for 90 successive days (normal control, named C). Group 2, rats fed high fructose diets for 90 successive days (obese rats, named HFFD) [26]; Group 3, rats fed HFF-diet and received 200 mg/kg of body daily for 90 successive days (HFFD + EAWE); while Group 4, rats fed HFF-diet and received 5 mg/kg of atorvastatin daily for 90 days by gastric gavage route as described by our previous study [26] (HFFD + Atorv). At the end of the study, the rats were weighted using a digital weighing scale, sacrificed by decapitation. The blood was collected after decapitation and the serum were stored at -80 °C until biochemical analysis. The intestine of each rat was excised and the lumen was flushed out in 0.9% NaCl buffer. The pancreas and the intestine mucosal tissue were pooled, homogenized, and centrifuged at 5000×*g*. The supernatant was conserved at -80 °C until lipase and α-amylase assays [26].

#### 2.3.4 Evaluation of toxicity of extract on rats

EAWE was administered by gavage, at a dose from 100 to 800 mg/kg daily to male rats. The rats are monitored every 4 h during the 7 days after administering the EAWE or saline buffer. The parameters were monitored: response to tail touch and grip. Physiological reflexes activities and response towards: ptosis, salivation and piloerection. The water and feed consumption and body weight Are monitored daily [32,33].

The article "Ephedra alata subsp. alenda (Ephedraceae) leaf extracts: phytochemical screening, anti-diabetic, anti-obesity and anti-toxic activities on diabetic-induced liver-kidney-testes toxicities and inhibition of α-amylase and lipase enzymes" was retracted in 2024. Reasons: concerns about the data; concerns about a third party's involvement.

#### 2.3.5 Biochemical analysis

The α-amylase activity was measured by the calculation of the rate of glucose obtained from CNPG3 substrate. A mixture of 20 μL of serum and 1 mL of CNPG3 was incubated at 37 °C for 5 min. The absorbance was measured at 405 nm (Kits Biomaghreb, Tunisia, ref 20033). Serum glucose level was determined by mixing 10 *μ*L of sample and 1 mL of glucose reagent, and then quinoneimine release was measured at 505 nm spectrophotometrically (Jenway 6405 UV/Visible, Great Britain) (Kit Biolabo France, ref 26019). The lipase activity was measured by colorimetric method. lipase activity leads to quinoneimine colored complex release was measured at 550 nm [34] (Kits, Biolabo, France, ref 99891). Total cholesterol (TC), Triglycerides (TG) and HDL-C levels were measured mixing 10 *μ*L of sample and 1 mL of reagent, which lead to pink colored quinoneimine and 4-Aminoantipyrine measured at 500 nm [35] (Kits, Biolabo, France, ref 80106, 80019 and 90206). LDL-C was quantified by calculating the difference between TC and HDLC values. Liver and muscles glycogen level was calculated according of the method described previously [36].

#### 2.3.6 Histological analysis

For histological examination, fragments of liver, kidney and testes were fixed in formaldehyde 10% and embedding into paraffin wax [37]. finally, liver, kidney and testes organ were sectioned into 5 μm-thick histological sections. Liver, kidney and testes sections were stained with hematoxylin and eosin solution (H &E), and photographed by a Olympus CX41 light microscope [18].

### 2.4 Statistical analysis

The values of each analysis were entered in StatView 5.0 for statistical analysis. One-way analysis of variance (ANOVA) and Fisher test was used to determine the significant variations (P < 0.05). All results, in this study, were presented as mean ± SD.

## 3 Results

### 3.1 Phytochemicals determination by HPLC-DAD analysis

Eight compounds were identified in *Ephedra alata* leaves extracts. Results of this study revealed both EAME and EAWE contain high quantity on cafeic acid (15 and 17%) and apigenin 7-O-glucoside (20 and 13%). A highest amount of apigenin 7-O-glucoside, rutin, p-Coumaric acid and cafeic acid contents (20,18, 17 and 15% respectively) in EAME, while the quantity of apigenin, luteolin-7-O-glucoside and gallic acid was higher in aqueous extract (12, 8 and 6% respectively) than that in methanolic extract. Vanilic acid was present in a small quantity in both EAWE and EAME. In addition, The HPLC–DAD analysis of the ethyl acetate of *Ephedra alata* leaves revealed the presence of two major phenolic compounds: Quercetin (57%) and apigenin (12%) **(**Table 1**,** Figure 1**).**

The article "Ephedra alata subsp. alenda (Ephedraceae) leaf extracts: phytochemical screening, anti-diabetic, anti-obesity and anti-toxic activities on diabetic-induced liver-kidney-testes toxicities and inhibition of α-amylase and lipase enzymes" was retracted in 2024. Reasons: concerns about the data; concerns about a third party's involvement.

**Table 1:** Phenolic compounds identified by HPLC-DAD analysis in aqueous extract (EAWE), methanolic extract (EAME) and ethyl acetate (EAEA) of *Ephedra alata* leaves.

Peak compound	RT (mn)	Compounds	UV spectrum λ_max_ (nm)	EAWE (%)	EAME (%)	EAEA
1	4.95	Gallic acid	280, 320	6	2	
2	12.49	Cafeic acid	220, 245, 325	17	15	
3	13.10	Vanilic acid	260, 295	4	3	
4	13.61	Rutin	218, 254, 352	9	18	
5	14.03	luteolin 7-O-glucoside	240, 265, 345	8	6	
6	14.27	p-Coumaric acid	234, 308	7	17	
7	15.92	Apigenin 7-O-glucoside	230, 275, 331	13	20	
8	18.82	Apigenin.	235, 270, 335	12		12
9	19.49	Quercetin	245, 370			57

**Figure 1:** HPLC chromatogram of water(A) methanol (B) andethyl acetate (C) extracts from leaves of *EA*.

### 3.2 In vitro experiments

#### 3.2.1 Effect of EAME, EAWE and EAEA on lipase activity

Table 2 showed the potential ability of EAWE to control obesity and hypercholesterolemia by inhibiting intestinal and pancreatic lipase activities. This study investigates that EAWE inhibited lipase activity with IC_50_ value 1.07 ± 0.09 mg/ml. The inhibitory activity of EAWE against lipase activity was 1.59 and 1.76-fold higher than EAME and EAEA respectively (**Tab.**

**Table 2:** : EAME, EAEA and EAWE lipase and α-amylase inhibition activity (IC50, mg/mL) (n = 3).

*Ephedra alata*	*IC*_*50*_*(mg/mL)*	
	α-amylase	Lipase
EAME	1,1 ± 0.12	1.71 ​± 0.14
EAEA	1,3 ± 0.1	1.89 ± 0.11
EAWE	0.39 ± 0.07	1.07 ​± 0.09
Acarbose	0.13 ± 0.03	
Atorvastatin		0.89 ± 0.07

#### 3.2.2 Effect of EAME, EAWE and EAEA on α-amylase activity

Table 2 showed that EAWE inhibited α-amylase activity *in vitro* with IC_50_ value: 0.39 ± 0.07. The IC50 values of EAME and EAEA were 1,1 ± 0.12 and 1,3 ± 0.1 mg/mL, respectively.

### 3.3 In vivo experiments

#### 3.3.1 Evaluation of the toxicity of EAME, EAWE and EAEA

This study observed that the administration of EAWE, EAME or EAEA to rats did not provoke any toxicity or perturbation up to a dose of 0.8 g/kg. EAME, EAWE and EAEA by the absence of any signs of toxicity and abnormalities as behavioral and physical changes; body weight variations and mortality. In this study, In the acute toxicity test, the of the EAWE, EAME or EAEA, at dose of 800 mg/kg, did not cause any death or physiological toxicity to the control group. EAWE, EAME or EAEA-treated rats presented no statistical variation in weight gain (P = 0.92), food (P = 0.96) and water (P = 0.97) consumption.

The article "Ephedra alata subsp. alenda (Ephedraceae) leaf extracts: phytochemical screening, anti-diabetic, anti-obesity and anti-toxic activities on diabetic-induced liver-kidney-testes toxicities and inhibition of α-amylase and lipase enzymes" was retracted in 2024. Reasons: concerns about the data; concerns about a third party's involvement.

#### 3.3.2 Effects of EAWE on food-water intake and body weight gain

Figure 2 showed that the mean daily food and water consumption were significantly (P < 0.01) increased in all HFFD rats compared to controls and this leads to significant (P < 0.01) increase of weight gain by around 44% (Figure 2C). The supplementation of EAWE to HFFD rats, during 3 months, significantly decreased food and water intake by 28 (P < 0.01) and 21% (P < 0.01) (Fig 2A, B) as compared to untreated HFFD-rats. Moreover, EAWE decreased the body weight by 12.6% (P < 0.05) (Figure 2C) as compared to untreated obese rats (Figure 2).

**Figure 2:** Average food intake (g/rat) (A), average water intake (ml/rat) (B); and body weight gain (C).

#### 3.3.3 Lipase activity and serum lipid rate of HFFD-rats treated with EAWE

In the obese rats showed a significant (P < 0.001) increase in the intestinal (Figure 3B) and pancreatic (Figure 3A) lipase activity in the obese rats by 107 and 222% respectively as compared to untreated obese rats. The increase in the lipase activity increased lipid digestion and, therefore distinguished increases in the serum total and LDL cholesterol rates by 19 (P < 0.05) and 68% (P < 0.01), respectively as compared to that of the normal rats. The supplementation of EAWE to obese rats was, however, decreased significantly (P < 0.01) the lipase activities in the intestine and pancreas by 33 and 36% respectively. Also, supplementation of EAWE to obese rats decreased TC and LDL-C by 18 (P < 0.05) and 34% (P < 0.01); and increased HDL-C by 27% (P < 0.01) in the serum (Table 3, Figure 3).

**Figure 3:** Effect of EAWE and obesity on pancreas (A) and intestine (B) lipase activities. ∗p < 0.05 as compared to normal rats; #p < 0.05 as compared to obese rats; ^@^p < 0.05 as compared to EAWE obese treated rats.

**Table 3:** Average food intake (g/rat), average water intake (ml/rat); and serum TC, LDL-C, and HDL-C rates in EAWE obese treated rats.

	Control rats	HFFD-rats	HFFD-rats + EAWE	HFFD-rats + Atorv
Average food intake (g/rat)	19.1 ± 2.3	26.3 ± 3.1	24.1 ± 2.7	22.1 ± 2.2
	16.3 ± 2.1	22.1 ± 2.7	19.3 ± 3.1	18.7 ± 2.1
TC (g/L)	0.63 ± 0.09	0.75 ± 0.10∗	0.61 ± 0.09#	0.69 ± 0.11#
HDL-C (g/L)	0.29 ± 0.03	0.19 ± 0.07∗	0.27 ± 0.11#	0.23 ± 0.06∗#@
LDL-C (g/L)	0.28 ± 0.02	0.49 ± 0.12∗	0.34 ± 0.13∗#	0.36 ± 0.07∗#@

The values are statistically presented as follows:

∗ p < 0.05 vs. normal rats.

# p < 0.05 vs obese rats.

@ p < 0.05 vs. obse EAWE obese treated rats.

#### 3.3.4 Effect of EAWE on α-amylase activity and serum glucose concentration

Obese rats showed an important increase in the intestinal (Figure 4B) and pancreatic (Figure 4A) α-amylase activity by 95 (P < 0.01) and 173% (P < 0.001) respectively in the obese rats. However, the supplementation of EAWE to obese rats suppressed the activity of this enzyme in the intestine and the pancreas, and decreased significantly (P < 0.01) the serum glucose rate (Figure 4C) by 20.8% as compared to untreated obese rats (Figure 4).

The article "Ephedra alata subsp. alenda (Ephedraceae) leaf extracts: phytochemical screening, anti-diabetic, anti-obesity and anti-toxic activities on diabetic-induced liver-kidney-testes toxicities and inhibition of α-amylase and lipase enzymes" was retracted in 2024. Reasons: concerns about the data; concerns about a third party's involvement.

**Figure 4:** Effect of EAWE and obesity on pancreas (A) and intestine (B) α-amylase activity, serum glucose level (C) and oral glucose tolerance test (D). ∗p < 0.05 as compared to normal rats; ^#^p < 0.05 as compared to obese rats; ^@^p < 0.05 as compared to EAWE obese treated rats.

#### 3.3.5 Effect of EAWE on OGTT

This study showed that the supplementation of 2 g/mL glucose to the normal rats caused an increase in the blood glucose level to a maximum of 1.83 g/L (P < 0.01) after 60 min and to return to normal value after 150 min. The administration of 2 g/mL glucose solution to obese rats induced a significant increase in serum glucose rate, with peak of 3.51 g/L (P < 0.001). The administration of EAWE, on the other hand, reduced the serum glucose peak to 2.01 g/L (Figure 4D).

#### 3.3.6 Effect of EAWE on liver and muscle glycogen rate

Liver and muscles of obese rats showed a significant (P < 0.001) decrease in the glycogen level in the liver (Figure 5A) and muscles (Figure 5B) of untreated obese rats. The supplementation of EAWE to HFFD rats increased significantly (P < 0.01) the glycogen rate in liver and muscle by 38 and 60% as compared to the control obese rats.

**Figure 5:** Effect of EAWE and obesity on liver (A) and muscle glycogen level (B). ∗p < 0.05 as compared to normal rats; #p < 0.05 as compared to obese rats; ^@^p < 0.05 as compared to EAWE obese treated rats.

#### 3.3.7 Effect of EAWE on obesity induced liver tissues toxicity

Liver of the obese rats showed histopathological alterations showed by the presence of portal inflammation and lymphocytic sinusoidal infiltration compared to normal control. In EAWE-treated obese rats, portal inflammation and lymphocytic infiltration were markedly reduced all liver tissues alterations (Figure 6).

**Figure 6:** Effect of EAWEadministration on HFFD-induced liver injury. C: Normal rat liver tissues. D: liver of Diabetics' rats: apparition of lymphocytic infiltrate in the portal and sinusoidal spaces. O + GAWE: HFFD-rats treated with EAWE; positive effect was observed evidenced by the absence of liver-infiltrating lymphocytes (H&E 100).

#### 3.3.8 Effect of EAWE on obesity induced kidney lymphocytes infiltration

Kidneys of the obese rats showed alteration of collecting system and interstitial lymphocytic infiltration when compared to normal rats. In EAWE-treated obese rats showed by the absence of all detected alterations (Figure 7).

The article "Ephedra alata subsp. alenda (Ephedraceae) leaf extracts: phytochemical screening, anti-diabetic, anti-obesity and anti-toxic activities on diabetic-induced liver-kidney-testes toxicities and inhibition of α-amylase and lipase enzymes" was retracted in 2024. Reasons: concerns about the data; concerns about a third party's involvement.

**Figure 7:** C: Normal rat kidney. O: diabetes provoked alteration in renal tissues. such as inflammation. D + EAWE: administration of EAWE to HFFD rats seems to have reverted all these histological toxicities (H&E 100).

#### 3.3.9 Histological alteration in testes obese rats treated with EAWE

Testes of obese rats showed a reduction of germ cells at various stages of development and somniferous tubules was showed in the testes of obese rats as compared to normal rats. In EAWE-treated obese rats, sperm abundance is normal and similar to those normal rats (Figure 8).

**Figure 8:** Effect of obesity on the histologicalmorphology of rat testes (magnification: ×100). C:Control ratsshowing a regular course of spermatogenesis. O: obese ratsviewing decrease in sperm count in somniferous tubules In EAWE-treated rats, spermatogenesis proceeded normally and somniferous tubules sperm count was near to that normal ratsgerm cells.

## 4 Discussion

Results of this investigation showed that HFF-diet for 12 weeks increased significantly pancreas and intestine lipase activity, body weight gain and altered serum lipid profile which is in agreement with previous reports [26,[38], [39], [40], [41], [42], [43]]. These studies revealed that HFFD could induce obesity by several mechanisms. A increase in lipase activity; and LDL and TG levels and decrease in HDL-C level in rat; that may be due to a decrease in the lipase activity, and consequently fat accumulation and therefore overweight and obesity [[44], [45], [46]]. Obesity caused by excessive fat and fructose consumption and lack of exercise. Excessive fat absorption and accumulation leads to the appearance of obesity [26,29,32]. Actually, one of the approaches to preclude hyperlipidemia, hypercholesterolemia, overweight, obesity and coronary artery diseases is the inhibition of free fatty acid and TG absorption in the small intestine and this by inhibition of lipase activity [6,30,47]. Therefore, inhibition of lipase activity in the intestine and pancreas is one of the most approach for the obesity [27]. This study evaluated the effect of EAWE, EAME and EAEA extracts on lipase activity. The IC50 value of EAME, EAWE and EAEA were 1.7, 1.07 and 1.8 mg/ml respectively; while the IC50 value for was 0.89 mg/ml (Table 2). This significant anti-lipase activity of EAWE is probably due to the presence of a variety of bioactive molecules as compared to EAME and EAEA. In fact, HPLC-DAD analysis revealed the presence of eight phenolic compounds namely cafeic acid, apigenin 7-O-glucoside, apigenin, rutin, luteolin 7-O-glucoside, p-Coumaric acid, gallic acid and vanilic acid (Table 1). Similarly, Danciu *et al* [48] have reported the presence of gallic acid, rutin, quercetin and its derivates in the EA extract. The most drugs evidenced in the EAWE could be involved in the inhibition of lipase activity et therefore anti-hyperlipidemia and anti-obesity effects. Recent previous investigations have shown that there is a positive correlation between food rich-flavonoids and polyphenols and obesity and type-2 diabetes prevention [6,31].

The article "Ephedra alata subsp. alenda (Ephedraceae) leaf extracts: phytochemical screening, anti-diabetic, anti-obesity and anti-toxic activities on diabetic-induced liver-kidney-testes toxicities and inhibition of α-amylase and lipase enzymes" was retracted in 2024. Reasons: concerns about the data; concerns about a third party's involvement.

In rats study, our results showed that supplementation of EAWE to obese rats decreased the intestinal and pancreatic lipase activity by 35 and 36% respectively as compared to untreated obese rats. The inhibitory effects of EAWE on intestinal and pancreatic lipase activity decreased significantly TC and LDL-C levels; and increase in HDL-C rate in the serum of obese rats. Also, the administration of EAWE to obese rats decreased significantly the body weight. The anti-obesity effect of EAWE is probably due to the presence of a variety of bioactive molecules evidenced by HPLC-DAD analysis (Table 1). According to the previous studies [48,49], the screening evidenced the presence of various phenolic compounds in the EA extracts such as cinnamic acid, apigenin-8-C-glucoside and epicatechin, Quercetin-3-O-glucuronide.

In fact, caffeic acid exists in EAWE a high percentage (17%) exerts a variety of pharmacological activities as the prevention of atherosclerosis and the anti-hyperglycemic activity through inhibition of α-amylase activity, stimulation of insulin secretion and prevention of insulin resistance [50,51]. Recently, Mu *et al* [51] have reported that dody weight gain, adipose tissue weight, TC and TG blood levels were significantly suppressed in the caffeic acid-treated rats.

Our study showed that apigenin is a flavonoid exists in EAWE a 12%. Gentile *et al* [52] have reported that in mice fed with HFD, the administration of apigenin decreased the body and epididymal fat weight and reduced the elevations of blood total cholesterol, triglycerides and glucose. Moreover, apigenin exerts an anti-diabetique effect by the decrease of the activity of the enzymes responsable of insulin resistance, and hepatic gluconeogenic enzymes activities and protect from liver and kidney dysfunctions and toxicities [53,54].

In addition, gallic acid presents with 6% decreased body weights in obese rats in according to previous studies. This therapeutic action can either be directly by inhibiting accumulation of lipid adipose tissue and liver, as well as directly by reducing lipase activity in intestine [55,56].

According of the study of Hsu *et al*, [57], the administration of rutin and coumaric acid to HFD rats for 8 weeks increased body organ weights, and suppressed epididymal adipose tissue weight.

The article "Ephedra alata subsp. alenda (Ephedraceae) leaf extracts: phytochemical screening, anti-diabetic, anti-obesity and anti-toxic activities on diabetic-induced liver-kidney-testes toxicities and inhibition of α-amylase and lipase enzymes" was retracted in 2024. Reasons: concerns about the data; concerns about a third party's involvement.

In addition, Mani *et al* [58] have reported that the oral nourishing of p-coumaric acid significantly suppressed the blood glucose rate in obese rats by the activation of the peripheral AMPK pathway [59] and the mTOR/S6 kinase pathway [60].

Obesity caused various complications such type-2 diabetes [26]. In fact, α-amylase is able to hydrolyze starch into disaccharides as maltase and sucrase [6,61,62]. This study investigated that water, methanol and ethyl acetate *Ephedra alata* extracts repressed α-amylase *in vitro* activity with IC50 0.39, 1.1 and 1.3 mg/ml respectively. This inhibitory effect of EAWE of α-amylase activity of EAWE is maybe due to the presence of a variety of bioactive compounds as cafeic acid, apigenin, rutin, p-Coumaric acid, gallic acid, vanilic acid… (Table 1). In obese rats, the supplementation of EAWE significantly reduced the intestinal α-amylase activity and this decreased in serum glucose rate by 34% as compared to control obese rats. The powerful inhibitory action of this digestive enzyme may be influenced by the presence of a variety of bioactive compounds in EAWE such as cafeic acid (17%), apigenin (12%), rutin (9%), p-Coumaric acid (7%) and gallic acid (6%) (Table 1). Theses bioactive compounds in EAWE can be useful in prevention of obesity and type 2 diabetes. Furthermore, EAWE was shown to be rich in phenolics content. HPLC-DAD) analysis of EAWE revealed the presence of cafeic acid (17%), apigenin (12%), rutin, which are largely responsible for various medicinal properties including anti-hyperglycemic effect. Oboh *et al* [63], have shown that flavonoids is a function of a specific pattern of their OH groups inhibited α-amylase. Ademiluyi *et al* [64] demonstrated that luteolin induce an inhibiting effect on α-amylase activity.

Hyperlipidemia and hyperglycemia are related to liver and kidney tissues damage, inflammation and dysfunctions. This study indicates that the administration of EAWE to obese rats protects from liver, kidney and testes toxicities. This protection may be due by the anti-hyperlipidaemia and anti-hyperglycaemia activities of EAWE. Similarly, Sioud *et al* have reported that *Ephedra alata* protects from liver and kidney toxicities [65]*.* The effect being attributed to a caffeic acid, apigenin and gallic acid^.^ The anti-hyperlipidemic and anti-hyperglycemia activities of EAWE may have protects from testes toxicity. In addition, Bourgou *et al* [66] have reported that EA extract Exerted a strong anti-inflammatory potential by the modulation of the secretion levels of inflammatory nitrite; and consequently protection of liver, kidney and testes from diabetes induced-inflammation [[67], [68], [69]].

The article "Ephedra alata subsp. alenda (Ephedraceae) leaf extracts: phytochemical screening, anti-diabetic, anti-obesity and anti-toxic activities on diabetic-induced liver-kidney-testes toxicities and inhibition of α-amylase and lipase enzymes" was retracted in 2024. Reasons: concerns about the data; concerns about a third party's involvement.

Some of the Although, that EAWE administration by gavage route improves obesity, type 2 diabetes and lipid profile. However, this study has a few limitations.

1. Another limitation is that the present observation does not provide information on whether EAWE supplementation confers a benefit of improving insulin sensitivity and glucose-lipid metabolism in obese rats
2. Also, a clinical study is very interesting to validate these results.
3. In addition, further studies are required to isolate the active drugs have therapeutic effects against obesity and type 2 diabetes.

## 5 Conclusion

The anti-obesity and the antidiabetic activities of EAWE was investigated. The obtained results suggest that *Ephedra alata subsp. alenda* leaves aqueous extract exerts a pronounced effect against type 2 diabetes and obesity by reducing body weight, hyperlipidemia and hyperglycemia and by the protection liver, kidney and testes functions in obese rats. This study, therefore, recommends the use of the aqueous extract of *Ephedra alata subsp. alenda* leaves in the management of obesity, type 2 diabetes and hyperlipidemia.

## Declarations

### Author contribution statement

Saber Abdelkader Saidi; Turki M. Al-Shikh: Conceived and designed the experiments.

Khaled Hamden: Performed the experiments; Analyzed and interpreted the data; Contributed reagents, materials, analysis tools or data; Wrote the paper.

### Funding statement

This research did not receive any specific grant from funding agencies in the public, commercial, or not-for-profit sectors.

### Data availability statement

Data included in article/supp. material/referenced in article.

### Declaration of interest's statement

The authors declare no conflict of interest.

### Additional information

No additional information is available for this paper.
